# Prediction Model of Bone Marrow Infiltration in Patients with Malignant Lymphoma Based on Logistic Regression and XGBoost Algorithm

**DOI:** 10.1155/2022/9620780

**Published:** 2022-06-28

**Authors:** Yongfen Huang, Can Chen, Yuqing Miao

**Affiliations:** ^1^Department of Hematology, Yancheng First Hospital Affiliated Hospital of Nanjing University Medical School, Yancheng No. 1 Peoples' Hospital, Yancheng 224006, China; ^2^Department of Hematology, Xuzhou Medical University, Xuzhou 221004, China

## Abstract

**Objective:**

The prediction model of bone marrow infiltration (BMI) in patients with malignant lymphoma (ML) was established based on the logistic regression and the XGBoost algorithm. The model's prediction efficiency was evaluated.

**Methods:**

A total of 120 patients diagnosed with ML in the department of hematology from January 2018 to January 2021 were retrospectively selected. The training set (*n* = 84) and test set (*n* = 36) were randomly divided into 7 : 3, and logistic regression and XGBoost algorithm models were constructed using the training set data. Predictors of BMI were screened based on laboratory indicators, and the model's efficacy was evaluated using test set data.

**Results:**

The prediction algorithm model's top three essential characteristics are the blood platelet count, soluble interleukin-2 receptor, and non-Hodgkin's lymphoma. The area under the curve of the logistic regression model for predicting the BMI of patients with ML was 0.843 (95% CI: 0.761~0.926). The area under the curve of the XGBoost model is 0.844 (95% CI: 0.765~0.937).

**Conclusion:**

The prediction model constructed in this study based on logistic regression and XGBoost algorithm has a good prediction model. The results showed that blood platelet count and soluble interleukin-2 receptor were good predictors of BMI in ML patients.

## 1. Introduction

Malignant lymphoma (ML) is a group of white blood cells that originated in lymphoid tissue tumors. ML is one of the most rapidly growing malignant tumors globally, especially non-Hodgkin's lymphoma (NHL), accounting for nearly 3% of cancer diagnoses and deaths [1]. Although the incidence of lymphoma in China is relatively low compared with that in developed countries such as the United States and Japan, the incidence is increasing rapidly. The study shows that the incidence of lymphoma in China has risen to 8th place in men and 13th place in women [2]. Lymphoma cells often spread throughout the body through the lymphatic system, such as bone marrow, lung, and liver. Bone marrow is the most common site of extranodal involvement in ML patients, and the frequency of involvement varies with lymphoma subtypes [3]. The assessment of bone marrow status is a critical step in the initial examination of ML patients. The bone marrow infiltration (BMI) of ML patients will affect the disease stage and extrapolar involvement of patients [4]. In addition, previous studies have reported poor prognosis in patients with BMI, and BMI is clear evidence of disseminated disease [5]. Therefore, the assessment of BMI status in ML patients can provide critical information for treatment decisions.

Because lymphoma metabolically recognizes all nodular, solid organ, cortical bone, and bone marrow diseases, positron emission tomography (PET)/CT or PET/MRI is required to evaluate Hodgkin's and non-Hodgkin's lymphoma [6]. However, bone marrow status assessment cannot be completed entirely by noninvasive means of PET/CT or MRI in clinical practice. Still, it can only be achieved by invasive bone marrow examination, including blood smear, biopsy, and flow cytometry [7, 8]. Various differentiated cells such as lymphoid, erythroid, and myeloid cells can be seen in bone marrow smears. Morphological methods are often tricky to identify lymphoma cells, and immunohistological processes are time-consuming and expensive [9]. Soluble interleukin-2 receptor (sIL-2R) and lactate dehydrogenase (LDH) have been reported for ML diagnosis and prognosis [10], but there is no previous research on BMI diagnosis in ML patients. Therefore, developing a new prediction model based on laboratory indicators during the first diagnosis has important guiding significance for clinical practice.

The traditional prediction model is mainly constructed based on logistic regression [11]. Machine learning algorithms have unique advantages in dealing with complex interactions and nonlinear relationships between variables [12–14]. In recent years, the use of the XGBoost algorithm in medical treatment has also gradually increased [15, 16]. Therefore, in this study, the logistic regression and XGBoost algorithm prediction model based on laboratory examination indicators were established to predict the occurrence of BMI in ML patients.

## 2. Materials and Methods

### 2.1. Clinical Data

A total of 120 patients diagnosed with ML in the hematology department of our hospital from January 2018 to January 2021 were retrospectively selected. The inclusion criteria were as follows: (1) The diagnosis of lymphoma followed the diagnosis criteria in the lymphoma diagnosis and treatment guidelines of the Chinese Society of Clinical Oncology [17]. (2) The bone marrow involvement was confirmed by immunohistochemistry, flow cytometry, and morphological examination. (3) The patient was generally in good condition, and the data of laboratory indicators were sufficient. Exclusion criteria are as follows: (1) patients during lactation/pregnancy, (2) patients > 80 years old, and (3) patients with other diseases of the blood system.

The staging of lymphoma in this study mainly referred to the lymphoma diagnosis and treatment guidelines of the Chinese Society of Clinical Oncology. The diagnostic criteria for lymphoma infiltrating bone marrow are as follows: Based on the classification of patients' bone marrow smears, when ≥5% of lymphoma cells are present in their bone marrow smears, or Reed-Sternberg cells are found, it is defined as bone marrow involvement by malignant lymphoma (ML-BMI).

### 2.2. Laboratory Prediction Index

Clinical baseline data, including gender, age, histological features, and laboratory indicators, were collected. Red blood cell count (RBC), hemoglobin (Hb), red blood cell distribution width (RDW), platelet distribution width (PDW), white blood cell count (WBC), platelet count (PLT), and platelet distribution width (PDW) were measured by automatic hematology analyzer. C-reactive protein (CRP) and erythrocyte sedimentation rate (ESR) were measured using an automatic CRP analyzer and an ESR, respectively. In addition, the examinations also include biochemical examinations, such as D-dimer (DD), CA153, CA125, *β*2-MG, alkaline phosphatase (ALP), and sIL-2R.

### 2.3. Construction of Prediction Model

Logistic regression is a commonly used method in machine learning to build a model that can distinguish two or more categories of samples. The logistic regression model is also common for credit data statistical analysis. Its essence is a linear regression model, and its core content is to study the relationship between dependent variables and multiple independent variables. A common form of logistic regression is the posterior probability expressed as category 0:

(1) $$\begin{array}{c} \mathrm{Pr}\left(Y=0\left|X=\chi \right.\right)=\sigma \left(\chi w^{T}\right)=\frac{1}{1+e^{-xw^{T}}}. \end{array}$$

The *Y* represents the category, *x* ∈ *R*_*f*_ represents the feature, *w* ∈ *Rf* represents the weight vector to be learned in model training. *σ* (*t*) = 1/(1 + *e*^−*t*^) is the sigmoid function that converts *xw*^*T*^ to posterior probability.

In machine learning, the loss function is used to measure the degree of agreement between the predicted value and the real value of the model. The smaller the loss function, the better the model. For logistic regression, the maximum likelihood estimation method is used to obtain the loss function:

(2) $$\begin{array}{c} J\left(w\right)=-\frac{1}{n}\overset{n}{\underset{i=1}{\sum }}\left[y_{i}\log\sigma \left(x_{i}w^{T}\right)+\left(1-y_{i}\right)\log\left(1-\sigma \left(x_{i}w^{T}\right)\right)\right]. \end{array}$$

In this formula, *n* is the number of samples.

The XGBoost is an iterative decision tree algorithm, which uses residuals to improve the model. Internal regularization can prevent overfitting and ensure the robustness of the model. First, XGBoost supports parallel computing, which calls all the cores of your computer to run simultaneously. Second, it also supports regularization, which prevents model overfitting. In addition, XGBoost comes with its cross-validation and missing value handling mechanisms, providing the flexibility to support personalized objective functions and metrics. Target loss function of XGBoost algorithm is as follows:

(3) $$\begin{array}{c} L=\overset{n}{\underset{i=1}{\sum }}l\left(y_{i},{\hat{y}}_{i}^{\left(t-1\right)}+f_{t}\left(x_{i}\right)\right)+\Omega \left(f_{t}\right)+C. \end{array}$$

Then, Taylor's second-order expansion of the objective function is performed:

(4) $$\begin{array}{c} L=\overset{n}{\underset{i=1}{\sum }}\left[l\left(y_{i},{\hat{y}}_{i}^{\left(t-1\right)}\right)+g_{j}f_{t}\left(x_{i}\right)+\frac{1}{2}h_{j}f_{t}^{2}\left(x_{i}\right)\right]+\Omega \left(f_{t}\right)+C. \end{array}$$

Finally, the evaluation function of the tree structure is obtained. The smaller the value is, the smaller the error is:

(5) $$\begin{array}{c} L^{*}=-\frac{1}{2}\overset{T}{\underset{j=1}{\sum }}\frac{G_{j}^{2}}{H_{j}+\lambda }+\gamma T. \end{array}$$

### 2.4. Research Queue

A total of 120 patients with ML were randomly divided into a training set (*n* = 84) and a test set (*n* = 36). The training set was used to construct the prediction model based on the logistic regression and XGBoost algorithm, and the test set data was used to evaluate the prediction effect of the model. The specific modeling process is shown in Figure 1. In addition, the training set was divided into BMI group (*n* = 23) and non-BMI group (*n* = 61) based on lymphoma cell content (≥5%) or the presence of Reed-Sternberg cell in patients' bone marrow smears. All items and clinical data from laboratory test indexes were included as predictors. Then, the results of the predicted indicators were compared between the two groups to screen out the indicators with risk factors (Figure 2).

### 2.5. Statistical Analysis

The SPSS20.0 software was used for the statistical analysis of the data. All data are expressed as the mean ± standard deviation. Shapiro–Wilk tests were performed to determine the normality of the data distributions. Independent sample *t*-test was used to compare groups, and 2 test was used to compare counting data groups. The SPSS20.0 software was used for statistical analysis. *P* < 0.05 difference was statistically significant.

## 3. Results

### 3.1. Comparison of General Data between the Training Set and Test Set

In the training set (*n* = 84), 51 female patients and 33 male patients were found. The average age was 45 (30-69) years. Twenty-five patients had systemic symptoms such as fever, night sweats, and weight loss. There were 14 female patients and 22 male patients in the test set. The mean age was 46 (29-69) years. There were 10 cases with systemic symptoms. There was no statistically significant difference between the general information of patients in the training set and the test set (*P* > 0.05). The details are shown in Table 1.

### 3.2. Comparison of Laboratory Parameters between Patients in the Training Set

In the training set, ML patients were divided into BMI group (*n* = 23) and non-BMI group (*n* = 61) according to whether they had BMI. Compared with the non-BMI group, RDW, CRP, ESR, DD, LDH, ALP, *β*2-MG, TRF, CA153, CA125, and SIL-2R were significantly increased in the BMI group (*P* < 0.05). In contrast, PLT levels in the BMI group were significantly lower than those in the non-BMI group (*P* < 0.05). The specific results are shown in Figure 3.

### 3.3. Extraction of Essential Features

By introducing the laboratory indicators in training set into the prediction model, we get the critical feature score results through calculation. The first two essential characteristics for predicting BMI in ML patients were PLT and sIL-2R, respectively (Figure 4).

### 3.4. Evaluation of the Effectiveness of the Prediction Model

Receiver operating characteristic (ROC) results showed that the area under the curve of the logistic regression model for predicting the BMI of patients with ML was 0.843 (95% CI: 0.761~0.926). The area under the curve of the XGBoost model is 0.844 (95% CI: 0.765~0.937), as shown in Figure 5.

## 4. Discussion

ML is one of the most rapidly growing malignant tumors in the world. Studies of lymphoma patients have shown that about 40% of ML patients have lesions that infiltrate the bone marrow. However, the exact diagnosis of BMI in patients with ML usually requires bone marrow biopsy, which can increase the risk of local infection, bleeding, bone marrow necrosis, and other invasive tests [18, 19]. Thus, establishing a BMI prediction model based on the laboratory indicators of ML patients at initial diagnosis has important guiding significance for clinical practice.

In this study, a prediction model was established based on logistic regression and XGBoost algorithm to predict the occurrence of BMI in ML patients. The results showed that the top three indicators associated with BMI were sIL-2R, PLT, and NHL. Previous studies have found elevated sIL-2R levels in patients with hair-cell leukemia [20], and since then, serum sIL-2R levels have been detected in patients with diffuse large B-cell lymphoma and follicular lymphoma [21]. The correlation between the sIL-2R level and prognosis of lymphoma was confirmed. Among the patients enrolled in this study, the incidence of NHL was as high as 90%, and nearly 25% of ML patients developed BMI. In addition, the weight coefficients of blood routine indexes, such as RDW, Hb, CRP, and ESR, are also good predictors. Anemia is often observed in lymphoproliferative diseases and has been considered an important prognostic factor of NHL. This anemia may be related to impaired iron reuse due to bone marrow involvement and inhibition of erythropoiesis by inflammatory mediators [22]. In addition, the results of this study showed that the PLT of BMI patients was reduced, while the platelet distribution width and DD were increased. The results suggested that BMI has an impact on the function of the coagulation system, and malignant diseases are usually accompanied by active coagulation and hypercoagulation [23]. Malignant tumor cells can activate the coagulation function by releasing proinflammatory and proangiogenic cytokines or directly interacting with the natural vasculature and blood cells. This change finally leads to the disorder of the coagulation system. The DD is a unique degradation product of cross-linked fibrin and is elevated in many types of cancer [24].

The prediction model constructed in this paper also included biochemical laboratory indicators of ML patients in the calculation. The results showed that LDH, TRF, and *β*2-MG had a better predictive performance. Previous studies have demonstrated elevated LDH levels in many types of cancer, often associated with poor prognosis in cancer patients [25]. Malignant tumor cells use 5-10 times more glucose than cells in normal tissue and convert most of the glucose into lactic acid. Increased LDH ensures an extensive glycolysis metabolism, thus storing energy for tumor growth [26]. Serum ALP mainly comes from the liver and bone, while the BMI of ML patients will lead to the release of ALP in the bone, which will lead to the elevation of serum ALP level. In addition, *β*2-MG is an essential protein for cell proliferation and is often regarded as a tumor marker [27]. In this study, the training set was divided into BMI group and non-BMI group for comparative analysis. The results showed that the CA125 level of patients in the BMI group increased significantly. Our results are similar to the high expression marker of CA125 in metastatic tumors proposed by previous study [28].

The effectiveness of the prediction model is also analyzed. All the models have good predictive efficiency. However, the area under the curve of the XGBoost model (0.844, 95% CI: 0.765~0.937) is more significant than that of the logistic regression model (0.843, 95% CI: 0.761~0.926). The result reflects the XGBoost algorithm's unique advantages in nonlinear relations [29].

There are several limitations to our study. First, this research for the single-center small sample cross-sectional retrospective study needs multicenter and large sample prospective studies for further verification. In addition, the laboratory indexes' analysis is not enough, and no related indicators are stratified analysis.

## 5. Conclusions

In conclusion, the prediction model constructed in this study based on logistic regression and XGBoost algorithm has a good prediction model. The results showed that PLT and sIL-2R were good predictors of BMI in ML patients.

## Figures and Tables

**Figure 1:** Flow charts for model construction and prediction.

**Figure 2:** Flow chart of risk index screening for bone marrow involvement in malignant lymphoma patients.

**Figure 3:** Comparison of laboratory index between the BMI group and the non-BMI group. All the indexes showed significant differences (*P* < 0.05).

**Figure 4:** Weight graph of prediction index based on logistic regression and XGBoost algorithm.

**Figure 5:** Receiver operating characteristic curve of the prediction model.

**Table 1:** Comparison of general data of patients in training set and test set.

	Male	Age	Systemic symptoms	NHL
Training set	51	45.77	25	22
Test set	22	46.53	10	54
*t*/*χ*^2^	0.002	0.463	0.048	0.985
*P*	0.967	0.644	0.827	0.321

## Data Availability

The data used to support the findings of this study are available from the corresponding author upon request.
